This article has been retracted.

# Analysis of Main Movement Characteristics of Hip Hop Dance Based on Deep Learning of Dance Movements

**DOI:** 10.1155/2022/6794018

**Published:** 2022-05-23

**Authors:** Rui Lu

**Affiliations:** Sports Department, Guizhou University of Finance and Economics, Guiyang 550000, Guizhou, China

## Abstract

In order to explore the main action characteristics of hip hop dance, a deep learning recognition system based on dance action is proposed. The network is based on convolution, pooling, and full connection calculation in a convolutional neural network (CNN). On the one hand, the pixel information in the video frame is extracted as the network input feature in the spatial domain. On the other hand, in the time domain, in order to better represent the change characteristics of video actions, optical flow information is introduced, and the optical flow vector change of pixels in DT time is calculated by the pyramid algorithm (LK) as the time domain convolution feature. In order to evaluate the performance of the network, this article takes the recognition of dance movements as an example to test the application of the algorithm. The test dataset contains 101 fully identified dance movements. The test results show that the proposed algorithm is 10.90% higher than F1 of inception V3, and the recognition accuracy is 10.85% and 5.27% higher than that of inception V3 and 3D-CNN networks, respectively. For the problems and difficulties brought by single-mode video action recognition, a multimodal action recognition method is introduced to achieve better results based on a large number of training data. Different depth networks have different characteristics. CNN network pays more attention to the relationship between local information, so it is suitable for image recognition and detection tasks. The RNN network is expanded in the time dimension, so it is suitable for the modal information related to similar videos. Therefore, based on multimodal information and a depth neural network, a depth feature extraction and fusion method for multimodal information is designed. Different methods of feature extraction and fusion are tried in the experiment, and the experimental results are analyzed. It proves that the deep learning and recognition of dance movement can effectively explore the main movement characteristics of hip hop dance.

## 1. Introduction

At present, the research on artificial intelligence promotes the development of intelligent robots in human-computer interaction. If we can build a visual perception system on the intelligent robot and reproduce the behavior close to humans, the robot can have a certain action imitation ability. This has broad application prospects in robot flexible operation, children's education, and service [1]. The hip hop dance, which takes action imitation as the way to realize, can analyze the human posture through machine vision and then imitate human actions, so it does not need to prepare action instructions in advance and has the function of recording action sequence and strong interaction. At present, robot dance mainly has the following ways: the form of man-machine cooperation; imitating human actions; motion generation based on music features; other action generation methods such as reinforcement learning, genetic algorithm, and random generation. The implementation approach based on action imitation includes two steps: capturing the demonstrator's action and reproducing the action. At present, the key link of the presenter's motion capture is mostly completed through a professional motion capture system [1]. This motion capture system includes a variety of sensing devices, which can be divided into three categories: optical motion capture system, inertial motion capture system, and motion capture system based on computer vision. In the field of robot motion imitation and motion following, the most common is to use the Kinect sensor to analyze the human skeleton with depth information. Kinect belongs to the third type of motion capture system. Multiple lenses form a depth sensor, which can calculate the depth information of objects through a computer vision algorithm. There are also some studies on motion capture through other types of systems, such as the wearable device Xsens MVN [1]. However, Kinect and other sensing devices are expensive, and their recorded data form is also special and not universal.  Figure 1 shows the reliance on specialized motion capture equipment, which limits the scope of human-computer interaction. With the continuous development of information technology, human motion recognition has gradually become a widely used problem in computer vision. Video-based human motion recognition usually refers to the use of various image processing and recognition classification technologies to extract and analyze the features of video data input and then realize the purpose of recognizing people's actions in video, which has a wide range of uses. By applying human movement recognition technology to dance video movement recognition, dance movements can be accurately identified, compared with standard movements, and irregular movements of dancers can be identified and corrected, which is a new method to assist dance teaching [2].

## 2. Literature Review

Sonawane and others changed the traditional separate training and sequential combination of attitude estimation and action recognition and proposed a framework combining attitude estimation and action recognition. The accuracy of motion recognition reaches the first-class standard, and the attitude estimation is improved [3]. Zhang and others proposed at the British Machine Vision Conference (BMVC) conference in 2011 that compared with the apparent features, the performance of gesture-based features in video data and even data with serious noise is better than that of action recognition based on underlying representation. Pose-based motion recognition can solve the problem of “intraclass spacing” perplexing appearance feature recognition, especially the invariance of 3D skeleton pose in appearance feature and viewing angle. Using gesture-based feature representation greatly simplifies the learning of motion recognition itself, but the representation feature is more general than the gesture feature. Therefore, in order to achieve higher accuracy and achieve the universality of motion recognition methods, many researchers generally choose to combine the two features. The disadvantage is that pose-based motion recognition will bring high computational complexity [4–6]. Sato and others proposed the method of spatiotemporal tree set for action recognition, found hierarchical spatiotemporal trees from training data, and then established action models on these trees for action classification in the video. Using a hierarchical spatiotemporal tree to represent actions can make the middle-level feature representation actions more robust. However, the exponential search space makes it difficult to find frequent and discriminant tree structures. A brief action vocabulary is established through discriminant clustering, and then this action vocabulary uses other tree clustering and sorting tree mining methods to select the closely combined high discriminant tree pattern. Obviously, the establishment of action vocabulary and the discriminant tree will bring a lot of calculation. The semantic-based method is to extract the middle-level semantic features such as object, scene, and pose,so as to make full use of all the information in the video scene [7]. Descriptive features used by Choi and others include atomic action, object, and attitude. They modeled the symbiotic statistics between these descriptive features and called the symbiotic relationship “action base.” Then, an action can be represented as a weighted combination of these “action base” subsets. However, this method is only effective for action recognition in specific scenes. In natural scenes, the recognition accuracy is low due to the inaccurate or incomplete definition of attribute space. Because each type of feature has its own advantages and can not cope with it, in recent years, it has been more inclined to fuse multiple features in feature extraction and construction to form a new feature descriptor for action recognition [8]. Kong and others proposed a convolutional neural network descriptor based on attitude for action recognition. The descriptor integrates the motion information and static information of the motion trajectory of each part of the human body, which greatly improves the recognition efficiency. However, the selection of color representation is limited, and the role of color realization is different in different action categories. Although the feature fusion method improves the robustness of features, researchers ignore the relationship between features when selecting fusion features, and more low-level features are selected for fusion, which will produce a certain amount of feature information redundancy [9]. Duinker and others extracted human action shape information through Canny edge detection to represent action edge information and then achieved the purpose of human action recognition by matching similar edges [10]. They extended the traditional SFS (shape from silhouette) method, which is only suitable for static objects to objects with rigid body motion, further extended it to articulated objects to obtain the shape and motion information of various parts of the human body, and estimated the position of human joints by solving the simple motion constraint equation between articulated parts, so as to achieve the purpose of motion recognition. However, using the underlying feature method for action recognition will lead to the inability to obtain all the action edge contour information when the human action is blocked or the background is complex, and the impact of incomplete information on human action recognition is direct and huge, which will directly lead to action recognition errors [11].

Based on the current research, a deep learning recognition system based on dance action is proposed. The network is based on convolution, pooling, and full connection calculation in a convolutional neural network (CNN). On the one hand, the pixel information in the video frame is extracted as the network input feature in the spatial domain. On the other hand, in the time domain, in order to better represent the change characteristics of video actions, optical flow information is introduced, and the optical flow vector change of pixels in DT time is calculated by the pyramid algorithm (LK) as the time domain convolution feature. In order to evaluate the performance of the network, this article takes the recognition of dance movements as an example to test the application of the algorithm. The test dataset contains 101 fully identified dance movements.

## 3. Theoretical Basis

### 3.1. Deep Learning Algorithm

The convolutional neural network is the most commonly used deep learning network in the field of image processing. The structure of the network is shown in Figure 2, which mainly includes convolution, pooling, and full connection operations.

#### 3.1.1. Convolution Layer

Convolution is a common mathematical operation in the field of information processing. The convolution operation method in the discrete field is shown as follows:

(1) $$\begin{array}{c} \left(f\cdot g\right)\left[n\right]=\sum_{-\infty }^{\infty }f\left(m\right)g\left(n-m\right). \end{array}$$

The convolution operation in the discrete domain requires a reasonable choice of convolution kernel, which is usually a matrix. The schematic diagram of the convolution operation is shown in Figure 3.

In Figure 3, *W* is the convolution kernel used and a 3 × 3 dimension is used. A convolution kernel can enhance or hide the pattern of features and extract image features flexibly.

#### 3.1.2. Pool Layer

The pooling layer refers to selecting a local region to replace the complete region in the features obtained by convolution, and pooling realizes the filtering and selection of features [12]. Common pooling operations include maximum pooling and mean pooling. The operation method of mean pooling is shown in Figure 4.

For a convolutional neural network, the introduction of the pooling layer realizes the downsampling of image information, which can effectively simplify the network structure and prevent overfitting.

#### 3.1.3. Full Connection Layer

The end of the convolutional neural network is the full connection layer, which can synthesize the characteristics of the previous layer to obtain the classifier of the network.

The connection diagram is shown in Figure 5.

The operation mode of the full connection layer is similar to that of the traditional single hidden layer neural network. It connects the input layer to the hidden layer and the hidden layer to the output layer by connecting weight and bias. The calculation method is shown in the following formula:

(2) $$\begin{array}{c} \left[\begin{array}{c} A_{1}\\ A_{2}\\ A_{3}\\ A_{4} \end{array}\right]=\left[\begin{array}{ccc} W_{11} & W_{12} & W_{13}\\ W_{21} & W_{22} & W_{23}\\ W_{31} & W_{32} & W_{33}\\ W_{41} & W_{42} & W_{43} \end{array}\right]\times \left[\begin{array}{c} X_{1}\\ X_{2}\\ X_{3} \end{array}\right]+\left[\begin{array}{c} b_{1}\\ b_{2}\\ b_{3}\\ b_{4} \end{array}\right]. \end{array}$$

#### 3.1.4. Output Layer

With the help of a nonlinear function, the output of the full connection layer is transformed into the final output of the deep network. For a binary classification problem, a logistic function is usually selected. The softmax cross-entropy function is selected in this article, and its form is shown in the following formula [13]:

(3) $$\begin{array}{c} \text{loss}=\sum_{i}\sum_{c}y_{c}\cdot \;\log\left(ypred_{c}\right), \end{array}$$

where C represents the category of classification. When the output result is consistent with the actual category, *y*_*c*_=1.

### 3.2. Double Convolution Neural Network Based on Space-Time Domain

The feature extraction method in the spatial domain is consistent with the image information extraction method. In this article, the features in the time domain are identified by optical flow. In the cyclic neural network, optical flow reflects the change trajectory of pixels after the motion state of objects in space, which is widely used in motion detection. The acquisition methods are as follows.

At time *t*, for the spatial coordinate position point O (c, r), the pixel brightness of this point is I (*c*, *r*, *e*). In DT time, the point moves to a new position (*c* + dc, *r* + dr) in the next frame. At this time, due to the extremely short time, the brightness of this point exists in the relationship in the following equation [14]:

(4) $$\begin{array}{c} A\left(c,r,e\right)=I\left(c+dc,r+dr,e+de\right). \end{array}$$

The Taylor expansion is shown in the following:

(5) $$\begin{array}{c} \frac{\partial A}{\partial c}\frac{\Delta c}{Ve}+\frac{\partial A}{\partial c}\frac{\Delta c}{Ve}+\frac{\partial A}{\partial c}\frac{\Delta e}{Ve}=0. \end{array}$$

At this time, the optical flow equation of this point can be obtained, as shown in the following:

(6) $$\begin{array}{c} \frac{\partial A}{\partial c}V_{c}+\frac{\partial A}{\partial r}V_{r}+\frac{\partial A}{\partial e}=0. \end{array}$$

In equation (7), *V*_*C*_ and *V*_*r*_ are optical flow vectors. From this differential equation, the pyramid (LK) algorithm needs to be introduced to solve the optical flow vector. The 3 × 3 pixel area of size contains 9 optical flow tracks, which can be expressed as the following equation in the form of matrix:

(7) $$\begin{array}{c} A_{v}=b. \end{array}$$

The variables are shown in the following equations:

(8) $$\begin{array}{c} b=\left[\begin{array}{c} -I_{t}\left(q_{1}\right)\\ -I_{t}\left(q_{2}\right)\\ ...\\ -I_{t}\left(q_{9}\right) \end{array}\right],\\ v=\left[\begin{array}{c} V_{x}\\ V_{y} \end{array}\right],\\ A=\left[\begin{array}{cc} I_{x}\left(q_{1}\right) & I_{y}\left(q_{1}\right)\\ I_{x}\left(q_{2}\right) & I_{y}\left(q_{2}\right)\\ ... & ...\\ I_{x}\left(q_{9}\right) & I_{y}\left(q_{9}\right) \end{array}\right]. \end{array}$$

The following equation can be solved by equation (8):

(9) $$\begin{array}{c} \left[\begin{array}{c} V_{x}\\ V_{y} \end{array}\right]={\left[\begin{array}{cc} \sum_{t}I_{x}{\left(q_{t}\right)}^{2} & \sum_{t}I_{x}\left(q_{t}\right)I_{y}\left(q_{t}\right)\\ \sum_{t}I_{x}\left(q_{t}\right)I_{y}\left(q_{t}\right) & \sum_{t}I_{y}{\left(q_{t}\right)}^{2} \end{array}\right]}^{-1}\cdot \left[\begin{array}{c} -\sum_{t}I_{x}\left(q_{t}\right)I_{t}\left(q_{t}\right)\\ -\sum_{t}I_{y}\left(q_{t}\right)I_{t}\left(q_{t}\right) \end{array}\right],\\ v={\left(A^{T}A\right)}^{-1}A^{T}b,\\ A^{T}Av=A^{T}b. \end{array}$$

## 4. Experimental Methods and Results

### 4.1. Experimental Design

The movements of hip hop dance include different walking movements, running movements, and jumping movements, and the changes are very rich. Its movements are composed of bending and stretching movements, rotating movements, surrounding movements, swinging movements, and wavy twisting movements of joints such as head, neck, shoulder, upper limb, and trunk. Each different movement has different fitness effects, which can coordinate the movements of upper and lower limbs, abdomen and back, and head and trunk, exercise each link and part of the body independently, comprehensively stimulate the muscles of the body, and train the head, neck, chest, legs, and hip. Most of the movements are around the ring and small joints, so exercise the small joints and small muscle groups that the body generally does not frequently move [15]. In addition, hip hop dance can also cooperate with breathing and the rhythm of the upper body of the body. There are many head and hand movements. The tension and relaxation of hip hop dance alternate to cooperate with the coordination of hip hop dance practitioners. Its movements have great explosive power, and the movements are very coherent, which can train the practitioner's sense of music and dexterity. If the intensity of exercise is moderate, it can have the characteristics of aerobic exercise. Learners can not only improve cardiopulmonary function but also lose weight [16].

In order to evaluate the effectiveness of the model, experiments are carried out on the dance video action dataset. The parameters of the dataset are shown in Table 1. In this dataset, there are 101 categories of dance movements, the number of frames of video is 25 FPS, and the resolution is 320 × 240, and the time length of the video is between 2.31 and 67.24 s.

In order to measure the recognition accuracy of the model for dance movements, the evaluation indexes F1 and MSE commonly used in deep learning are used in this article. The definition of these two indicators is shown in the following equations:

(10) $$\begin{array}{c} MSE=\frac{\sum_{I=1}^{N}{\left({\text{target}}_{i}-{\text{output}}_{i}\right)}^{2}}{N},\\ F1=\frac{2\times P\times R}{P+R}. \end{array}$$

### 4.2. Simulation Results

In order to better measure the recognition effect of the model in this article on dance movements in the video, this article introduces two deep convolution networks that have been widely used in industry: inception V3 and 3D-CNN networks. Their respective network parameter settings are shown in Tables 2 and 3, respectively.

Table 4 shows the parameter settings of the two-way convolution network in this article, which adopts two identical convolution structures. Through the comparison in Tables 2–4, it can be found that the complexity of the three networks is basically the same. The video database given in Table 1 is divided into the training set and test set according to the ratio of 7 : 3 [17]. After three network training processes, the test set is used for testing. The test results are shown in Table 5.

It can be seen from the test results in Table 5 that among the three networks, the worst network F1 index is 69.32% of that of Inception V3, the middle is the 3D-CNN network, and the best is the two-way convolution network, which is 10.90% higher than that of F1 of Inception V3. MSE and F1 are two mutually negatively correlated indicators. The data in column 3 of Table 5 preferably verify this data trend and prove the effectiveness of the test results [6]. From the accuracy of dance action recognition in column 4 of Table 5, due to the introduction of manually extracted time domain optical flow information, the dual CNN algorithm proposed in this article has improved by 10.85% and 5.27% for Inception V3 and 3D-CNN networks, respectively.

For the UCF-101 video, from the first frame to the last frame, 16 frames are extracted from the current frame with a step of 1. This can effectively increase the scale of data and reduce the occurrence of overfitting. Therefore, the final input video stream size is 128 ∗ 171 ∗ 3 ∗ 16, corresponding to the length, width, number of channels, and video frame length of the video frame, respectively. The total attack of the network uses 8 convolution layers, 5 maximum pooling layers, and 2 full connection layers. Finally, Softmax is connected as the output layer. The convolution kernel size ranges from 64 in the lower layer to 512 in the upper layer, and the corresponding feature expression is also a process from general to special.

The training adopts the random gradient descent method to update the weight, and the learning rate is initially set to 0.01. The decreasing trend of loss in the final training process is shown in Figure 6. The vertical axis is the loss and the horizontal axis is the number of iterations.

For the recursive cyclic network used for bone point information, because the processed features obtained after preprocessing are enough to be used for training, there is no pretraining process. Finally, the structure of the stacked lstm-rnn network is used in this experiment. There are 512 hidden units in the two-layer rnn-lstm network, and 0.5 dropout is added to prevent overfitting. The network uses the random gradient descent optimization algorithm, the basic learning rate is 0.001, the momentum is 0.9, and the learning attenuation rate is 0.0005. The training process is shown in Figure 7.

Transfer learning is used to transfer the knowledge learned from the original database to new knowledge on similar datasets. With the emergence of transfer learning, researchers can get good training results when the amount of new datasets is small, the annotation is incomplete or small, and the distribution of training sets and test sets is different. For convolution neural networks, the representation of convolution kernel is a process from a low level to a high level, from general to special, so low-level features can also be used for similar tasks.

After training the 3D-CNN network through UCF-101, the pretraining model is obtained. Modify the final output K of the network as the number of categories of the database for fine-tuning. Take the MSR3D Online Action database as an example; the sample has 7 categories, so *k* = 7. In the process of fine-tuning, the learning rate is reduced to 0.0001 to adjust the parameters.  Figure 8 shows the fine-tuning training process of the 3D-CNN network, in which the horizontal axis is the number of iterations and the vertical axis is the network output loss.

After obtaining the static and dynamic features and probability of human behavior, we can achieve better results by fusing the two features. In this experiment, two methods of feature fusion are tried, which are called early fusion and late fusion.

In the early stage of fusion, the first fully connected (FC) layer of the 3D-CNN network and the FC-6 layer connected with the recurrent neural network are fused into a single feature by splicing or superposition as the overall feature of the input video. In the late fusion, the probability outputs of the 3D-CNN network and recurrent neural network are superimposed by linear weighting to obtain the final prediction value specifically as follows:

(1) The late fusion adopts the method of probability linear weighting:
  (11) $$\begin{array}{c} P=\frac{1}{N}\left(\sum_{i=1}^{N}\alpha P_{1}+\left(1-\alpha \right)P_{2}\right), \end{array}$$
where *α* is the weighting parameter, *P* and *P* are the probability of independent static information and dynamic information, respectively, and *P* is the final prediction probability.
(2) In the early fusion method, the final features are obtained by extracting the features of static and dynamic information, respectively, splicing the full connection layer of the two networks, or linearly superimposing the full connection layer features. In this experiment, the fusion features are classified by the SVM classifier.

Figure 9 shows the impact of parameter *α* on the final classification accuracy when late fusion is adopted to weight the probability of single feature classification in the feature fusion stage. When *α*-0.3, the classification accuracy is the highest, but it is still lower than that of late fusion feature reclassification.

Figure 10 shows the process of the three-dimensional convolution network in the pretraining stage and network fine-tuning stage, respectively, and the black and red broken lines are the function loss output of the pretraining and fine-tuning process, respectively. It can be seen that the fluctuation and loss output are large in the training process, and the network output loss is reduced after fine-tuning, so the final classification effect of the model is improved and the network learning time cost is reduced.

Firstly, this chapter introduces the action recognition method based on deep learning in a single mode, including a convolutional neural network and recursive neural network. It also explains the problems and difficulties brought by single-mode video action recognition, and introduces a multimodal action recognition method. Deep learning obtains better results based on a large number of training data. Different depth network characteristics are also different. CNN network pays more attention to the relationship between local information, so it is suitable for image recognition and detection tasks. The RNN network is expanded in the time dimension, so it is suitable for the modal information related to similar videos. Therefore, based on multimodal information and depth neural network, a depth feature extraction and fusion method for multimodal information is designed. Different methods of feature extraction and fusion are tried in the experiment, and the experimental results are analyzed.

In the process of learning and training, hip hop dancers should master the basic steps, first master the movements of the lower limbs, then learn the movements of the body and upper part, and control the movement synchronization of all parts of the whole body; that is, the movements of lower limbs are organically combined with those of trunk and upper limbs. In the learning process of aerobics, most of the movements are “horizontal and vertical,” so we should pay attention to the body shape, but hip hop dance emphasizes the randomness of movement, and the movements are very relaxed. Therefore, we should relax our muscles and joints in the practice process so they are more flexible and coordinated. Therefore, hip hop dance is generally performed under the weak beat of the soundtrack. The soundtrack selects *R*&B music, so the sense of rhythm is very strong. In the movement of hip hop dance, the body will form a very large rhythm, which will stimulate the spirit of learners and stimulate the emotion of dance practice. The action is very bright, enthusiastic, and energetic, so it is very in line with the needs of the times and is welcomed by young people.

## 5. Conclusion

In this article, the video action recognition methods are studied. Through the investigation of the traditional deep convolution networks, it is found that the features extracted by these deep networks are more spatial information and lack time domain information, which affects the accuracy of action recognition. In this article, the optical flow information is used to characterize the state changes of time domain movements, and a two-way convolution network is constructed, which greatly improves the recognition accuracy of dance movements. In the follow-up research, we can continue to optimize the structure of time domain convolution network and improve the performance of the algorithm. The soundtrack is *R*&*B* music, so the sense of rhythm is very strong. In the movement of hip hop dance, the body will form a very large rhythm, which inspires the spirit of learners and stimulates the emotion of dance practice. The action is very bright, enthusiastic, and energetic, so it is very in line with the needs of the times and thus, is welcomed by young people.

## Figures and Tables

**Figure 1:** System flowchart.

**Figure 2:** Convolutional neural network.

**Figure 3:** Schematic diagram of the convolution operation.

**Figure 4:** Schematic diagram of the mean pooling operation.

**Figure 5:** Schematic diagram of the whole connection layer.

**Figure 6:** Decreasing trend of pretraining network loss.

**Figure 7:** Training error diagram of recurrent neural network.

**Figure 8:** Fine-tuning process of 3D convolution network.

**Figure 9:** Influence of *α* value on the final result of network output.

**Figure 10:** Pretraining and fine-tuning of three-dimensional convolutional network loss.

**Table 1:** Dataset parameters.

Parameter name	Parameter value
Total number of categories	101
Total videos	13300
Average video duration	7.30 s
Total video duration	1600 min
Frame rate	25 fps
Resolving power	320 × 240

**Table 2:** Parameter setting of inception V3.

Layer name	Patch size	Input size
Conv1	3 ∗ 3/2	300 ∗ 300 ∗ 3
Conv2	3 ∗ 3/1	150 ∗ 150 ∗ 32
Conv padded	3 ∗ 3/1	148 ∗ 148 ∗ 32
Pool1	3 ∗ 3/2	148 ∗ 148 ∗ 64
Conv3	3 ∗ 3/1	74 ∗ 74 ∗ 64
Conv4	3 ∗ 3/2	72 ∗ 72 ∗ 80
Conv5	3 ∗ 3/1	36 ∗ 36 ∗ 192
3∗Inception	—	36 ∗ 36 ∗ 288
5∗Inception	—	18 ∗ 18 ∗ 768
2∗Inception	—	9 ∗ 9 ∗ 120
Pool2	9 ∗ 9	9 ∗ 9 ∗ 2048
Linear	Logits	1 ∗ 1 ∗ 2048
Softmax	—	1 ∗ 1 ∗ 500

**Table 3:** 3D-CNN network parameter settings.

Layer name	Patch size	Input size
Conv1	3 ∗ 3/2	300 ∗ 300 ∗ 3
Conv2	3 ∗ 3/1	150 ∗ 150 ∗ 32
Conv3	3 ∗ 3/1	148 ∗ 148 ∗ 32
Conv4	3 ∗ 3/2	148 ∗ 148 ∗ 64
Conv5	3 ∗ 3/1	74 ∗ 74 ∗ 64
Conv6	3 ∗ 3/2	72 ∗ 72 ∗ 80
Conv7	3 ∗ 3/1	36 ∗ 36 ∗ 192
Fe1	Logits	36 ∗ 36 ∗ 288
Fe2	Logits	18 ∗ 18 ∗ 768
Fe3	Logits	9 ∗ 9 ∗ 120
Linear	Logits	1 ∗ 1 ∗ 2048
Softmax	—	1 ∗ 1 ∗ 500

**Table 4:** Parameter setting of two-way convolution network.

Layer name	Patch size	Input size
Conv1	7 ∗ 7/2	224 ∗ 224 ∗ 2
Conv2	5 ∗ 5/2	117 ∗ 117 ∗ 96
Conv3	3 ∗ 3/1	56 ∗ 56 ∗ 256
Conv4	3 ∗ 3/2	14 ∗ 14 ∗ 512
Conv5	3 ∗ 3/1	14 ∗ 14 ∗ 512
Conv6	3 ∗ 3/2	14 ∗ 14 ∗ 512
FullConnect1	Logtis	7 ∗ 7 ∗ 512
FullConnect2	Logtis	1 ∗ 1 ∗ 2048
Softmax	—	1 ∗ 1 ∗ 500

**Table 5:** Performance comparison of three networks.

Model	F1 (%)	MSE	Recognition accuracy (%)
Inception V3	69.32	0.220	72.63
3D-CNN	74.21	0.172	77.94
Dual CNN	80.22	0.133	83.21

## Data Availability

No data were used to support this study.
